# Four Simultaneous Opportunistic Infections in a Man With Newly Diagnosed HIV

**DOI:** 10.7759/cureus.92629

**Published:** 2025-09-18

**Authors:** Kai Yoshinaga, Saipriya Ayyar, Adam Sanderson, Hari Polenakovik

**Affiliations:** 1 Internal Medicine, Wright State University, Dayton, USA; 2 Infectious Disease, Wright State University, Dayton, USA

**Keywords:** candida, cmv, hiv, hsv, pcp

## Abstract

Human immunodeficiency virus (HIV) directly inhibits the function of the immune system via its anti-CD4 T cell activity, and much of the morbidity associated with HIV is secondary to the effects of opportunistic infections. Advancements in both efficacy and accessibility of HIV screening and therapies have led to patients being managed earlier in their disease courses. This is the case of a 38-year-old male who initially presented with chest pain and was diagnosed with HIV in the setting of four simultaneous opportunistic infections.

## Introduction

In 2022, nearly 38,000 people received a new human immunodeficiency virus (HIV) diagnosis [1]. With increased screening, more advanced therapy, and more accessible and affordable antiretroviral therapies, fewer patients are now presenting with advanced HIV and opportunistic infections [2]. HIV infection directly affects the CD4 T cell count, thus limiting the immune system’s response to infection and increasing the risk of opportunistic infections. Early effects on CD4 T cell counts increase the risk of tuberculosis, while further decreases in CD4 T cell counts increase the likelihood of many other viral, bacterial, and fungal infections [3]. Progressive loss of CD4 T cell count leads to a corresponding increased threat of opportunistic infections in untreated HIV patients [4]. We present a rare case of a patient with routine care who presented to the hospital with four simultaneous opportunistic infections: esophageal candidiasis, *Pneumocystis jirovecii *pneumonia (PCP), human simplex virus-2 (HSV-2) perianal ulcers, and cytomegalovirus (CMV) esophagitis.

## Case presentation

The patient was a 38-year-old male with no significant past medical history who presented to the hospital for chest pain. In the three months leading up to admission, he had odynophagia with significantly limited oral intake, leading to over 20 pounds of weight loss. He stated that in the three days prior to admission, he had not been eating and had limited fluid intake. He also endorsed significant weakness, which he associated with the severely limited oral intake. He had a history of inhaled methamphetamine use but had not engaged in that activity in several years. After an initial extensive evaluation to rule out a cardiac etiology of chest pain, further discussions led to the patient reporting a history of unprotected high-risk sexual activity, penetrative and receptive, with multiple male and female partners. He was not screened for HIV previously. The patient then also endorsed several weeks of perianal pain. He denied any constitutional symptoms as well as any shortness of breath, abdominal pain, or diarrhea.

In the emergency department, his vitals were stable and within normal limits. The physical exam was significant only for oral thrush and perianal ulcers. Laboratory evaluation is presented in Table 1. 

**Table 1:** Laboratory tests completed with resulting values and reference ranges TIBC, total iron-binding capacity; CMV, cytomegalovirus

Lab Test	Value	Reference Range
Hemoglobin	9.0 g/dL	13-17 g/dL
WBC	5.6 k/uL	4.0-10.0 k/uL
Neutrophil (%)	85.90%	46-78%
Absolute neutrophil count	4790	~1.8-7.0 × 10³/µL
Lymphocyte (%)	9.60%	18-52%
Absolute lymphocyte count	538	~0.7-3.9 × 10³/µL
hsTroponin	3 ng/L	<22 ng/mL
Haptoglobin	287.8 mg/dL	0.47-2.1 g/L
Total iron	18 mcg/dL	65-180 mcg/dL
TIBC	152 mcg/dL	240-460 mcg/dL
Iron saturation (%)	11%	20-50%
Ferritin	1784.2 ng/mL	12-300 ng/mL
Hep B surface antibody	Positive	-
Hep B core antibody	Negative	-
Hep B surface antigen	Negative	-
HIV 1 antibody	Positive	-
HIV-1 RNA qPCR	2,050,000 copies/mL	-
HIV-1 subtype	B	-
CMV DNA qPCR	2767 IU/mL	-
HSV 2 PCR	Positive	-
1,3 Beta-D-glucan	>500 pg/mL	<60 pg/mL

An initial chest X-ray was notable for ill-defined increased lung markings in the perihilar regions bilaterally. A computed tomography (CT) of the chest on hospital day 3 found diffuse moderate to severe predominantly ground-glass attenuation in all lobes of the lungs (Figures 1, 2). Due to these findings, in conjunction with his 1,3 beta-D-glucan level, he was started on high-dose sulfamethoxazole-trimethoprim for PCP treatment. Due to HSV-2 PCR positivity, acyclovir was started. In addition, a single dose of micafungin followed by fluconazole was given due to oral and suspected esophageal candidiasis. He underwent esophagogastroduodenoscopy (EGD) with biopsies, which demonstrated an inflamed distal esophageal area with small patches of desquamated mucosa and white plaques (Figure 3) and oral thrush (Figure 4). Otherwise, the stomach and duodenum were without focal abnormalities. Pathology on the esophageal biopsies found acute ulcerative esophagitis with budding yeast and hyphae consistent with fungal esophagitis. Immunostaining was positive for rare CMV inclusions and negative for HSV. Acyclovir was replaced by valganciclovir to cover both HSV and CMV.

**Figure 1:** CT sagittal view at level of the primary bronchi demonstrating diffuse opacities

**Figure 2:** CT axial view demonstrating diffuse ground-glass opacities with peripheral sparing

**Figure 3:** EGD imagining of the distal esophagus with white plaques, from which cold biopsies were obtained and demonstrated CMV nuclear positive staining Arrows indicate locations of plaques. EGD, esophagogastroduodenoscopy; CMV, cytomegalovirus

**Figure 4:** EGD imaging with extensive oral thrush at the level of the uvula EGD, esophagogastroduodenoscopy

With appropriate treatments, the patient’s odynophagia began to improve, and he was feeling well for discharge. Upon discharge, the patient was continued on sulfamethoxazole-trimethoprim, valganciclovir, fluconazole, bictegravir, emtricitabine, tenofovir alafenamide, and a prednisone taper. At a follow-up appointment eight weeks later, the patient had a recurrence of his esophageal candidiasis with recurrence of odynophagia, which required additional treatment with a further two-week fluconazole course, but his other symptoms of fevers, weakness, and chest pain largely resolved.

## Discussion

This case of a gentleman with four simultaneous opportunistic infections is a rare first presentation of HIV in the era of advanced screening and readily available therapies. Since 2010, the incidence of people acquiring HIV has been reduced from 2.1 million to 1.3 million in 2023 [5]. Over the same time period, HIV-related deaths worldwide have been reduced from 1.3 million a year to 630,000 a year. In 2023, 86% of people living with HIV knew their HIV status, and that number is predicted to rise to 95% in 2025. Despite these reassuring statistics, screening is still an invaluable asset to the medical community in establishing early diagnoses for these patients. For instance, this patient had never undergone HIV testing despite his varied sexual partners and lack of barrier protection use. Approximately 80% of new HIV transmissions are from persons who do not know their HIV-positive status or are not receiving regular care [6]. While the presence of opportunistic infections in patients with diagnosed HIV is not uncommon, it is rare for a new diagnosis of HIV to be made due to multiple concurrent opportunistic infections, given recent diagnostic and therapeutic advancements. 

Patients with HIV are at increased risk of esophageal candidiasis and PCP at CD4 T cell counts <200, HSV-2 infections at CD4 T cell counts <100, and CMV infections at CD4 T cell counts <50. A meta-analysis performed in 2016 found the following incidences of acquired immunodeficiency syndrome (AIDS)-defining illnesses in antiretroviral treatment (ART)-naïve patients: esophageal candidiasis 3.0%, PCP 2.8%, and herpes simplex 6.0% [2]. Rates of CMV infection in immunocompromised patients are as high as 40%, and CMV esophagitis is the second most common manifestation of gastrointestinal CMV, after CMV colitis [7,8]. CMV esophagitis is diagnosed by the presence of ulcers in the distal esophagus with concomitant biopsy findings of intranuclear inclusion bodies [9]. Treatment of CMV involves induction with valganciclovir or ganciclovir followed by maintenance with valganciclovir, with eventual immune reconstitution being therapeutic. The presence of all four of these AIDS-defining illnesses puts this patient in a notable statistical minority of ART-naive patients. 

Oropharyngeal and esophageal candidiasis are common in patients with HIV infections [10]. There are no measures to reduce Candida exposure, given its ubiquitous presence on human mucosal surfaces, and primary prophylaxis is not recommended. Chronic suppressive therapy may be beneficial in patients with frequent or severe recurrences, but it is generally not recommended due to the effectiveness of acute therapy and the low mortality rate of mucocutaneous diseases [11,12].

*P. jirovecii* is a ubiquitous fungus, with most healthy individuals developing antibodies to it by the age of 2-4 years old [13]. PCP occurred in approximately 70-80% of patients with AIDS prior to the advent of PCP prophylaxis and ART and was associated with a 20-40% mortality rate in those with significant immunosuppression who were treated for PCP. Diffuse, bilateral, symmetrical ground-glass interstitial infiltrates in a butterfly pattern are common chest radiograph findings, while early in the disease process, a chest radiograph may be unremarkable. Beta-D-glucan is a polysaccharide present in the cell walls of Pneumocystis. Testing of beta-D-glucan has a pooled sensitivity/specificity of 95%/86% and a negative predictive value of over 95%. Sputum PCR and direct fluorescence analysis of sputum are more specific and definitive tests. Treatment typically involves sulfamethoxazole-trimethoprim with or without corticosteroids, depending on severity [14].

Infections with HSV-1 and HSV-2 are common in the United States, with HSV-1 seroprevalence of 47.8% and HSV-2 seroprevalence of 11.9%. Among HIV-infected individuals, approximately 70% are HSV-2 seropositive and 95% are seropositive for either HSV-1 or HSV-2. HSV-2 infection significantly increases the risk of HIV infection, and HSV-2 reactivation increases HIV RNA levels in the blood and genital secretions in co-infected individuals. HSV-1 most commonly manifests as orolabial herpes, typically characterized by a sensory prodrome in the affected area, followed by lesions that progress from papule to vesicle with ulceration and finally crust over on the lips and oral mucosa. Genital herpes is typically caused by HSV-2. Extensive, deep, nonhealing ulceration can occur in significantly immunosuppressed individuals. HSV DNA PCR and viral culture are the preferred methods for the diagnosis of mucocutaneous lesions.

## Conclusions

Several decades ago, HIV was one of the most deadly epidemics worldwide, but with advances in screening, diagnostics, and appropriate therapies, the morbidity and mortality of this disease have been progressively improving. While more individuals living with HIV know their status than ever before, the value of history taking cannot be overstated for the newly presenting patient who may not have been screened in the past, or may have contracted the disease since screening. We encourage providers to keep undiagnosed HIV with opportunistic infections on the differential in otherwise healthy presenting individuals. This patient, who presented with four concurrent opportunistic infections, demonstrates a rarity in an urban city environment with relatively robust and accessible healthcare.
